This article has been retracted.

# Enhanced Invisibility and Robustness of Digital Image Watermarking Based on DWT-SVD

**DOI:** 10.1155/2022/5271600

**Published:** 2022-01-28

**Authors:** Ali Alzahrani

**Affiliations:** Department of Computer Engineering, King Faisal University, Al-Ahsa, Saudi Arabia

## Abstract

The propagation of digital media over the Internet has helped improve digitization, which has given an excessive lead to copyright issues. Digital watermarking techniques have been applied to address copyright issues. In research, a system is being developed to handle veracious types of watermarked attacks, for obtaining extreme security and an adequate level of visibility and robustness. The discrete wave transform (DWT) and singular value decomposition (SVD) approaches were applied to analyze veracious types of attacks. The DWT method was used to embed the host image in four levels; this level was processed using the SVD method. The peak signal-to-noise ratio (PSNR) and structural similarity index measure (SSIM) were applied to measure the invisibility, and the normalization correlation (NC) was used to examine the robustness of watermarked images. The empirical results showed that the proposed DWT-SVD achieved superior accuracy in identifying the various attacks. The proposed DWT-SVD performance was confirmed during the training process, and the proposed system was shown to have high invisibility and robustness against various types of attacks on watermarked images. Finally, the results of the proposed system were compared to existing systems, and it was shown that DWT-SVD achieved better performance in terms of pixel-value modification attacks.

## 1. Introduction

Electronic document safeguarding was and remains one of the most critical problems in scientific investigation. With the development of Internet technologies, intruders are illegally duplicating, authenticating, and distributing digital materials. Watermarking technologies have thus been investigated for a variety of purposes, including broadcasting, tracking, intellectual property protection, document verification, and copying restriction [1]. With the extensive posting and distribution of electronic information on the Internet, breaches of copyrights, unauthorized usage, reproduction, and online content theft have become more common. Digital images represent high-value-added resources, which involve the protection of their intellectual property copyrights. However, digital watermarking [2] is considered a current and useful technology for protection of such images. Watermarking technique (WM) can be employed to encode the owner's data, which is then preserved or circulated on the Internet. This technique is used to assert proprietorship through retrieving the encoded watermark data when needed, as per the current technologies, applications fields, and other online platform-based systems. Limited studies have been investigated for digital watermarking images. Recently, different approaches have been be implemented to perform watermark embedding, and extracting the WM from the digital image algorithmically or changing it has been introduced [3–9]. Generally, watermarking may be subjected to a harmful attack aimed at destroying or removing the encoded WM data, as well as a nonmalicious attack through procedures that must be used to preserve or circulate the content. As a result, WM embedding could be accomplished in either an algorithmic or a mechanistic manner. WM extraction, on the other hand, has a different scenarios. The WM-incorporated host information may be destroyed as a result of malicious or nonmalicious cyberattacks, and the embedded WM data might be lost. As a result, extracting the WM programmatically or sequentially may well not be effective, and a statistical technique may provide better performance.

One or two merged watermark images can be formed through a sort of semisequence received from such a pseudorandom cryptographic security. A monochrome or unicolor image can be used as a watermark. Scattered spectral (SS) [10–12] and quantization index manipulation (QIM) [13] are two content protection systems for watermarking schemes, which are commonly characterized as cumulative and alternative, respectively. STDM (spread transform dither modulation) [14] is a type of QIM that is particularly resistant to requantization and external disturbance intrusions. STDM unites the reliability of SS with the efficiency of QIM. The payload, reliability, and authenticity of watermarking techniques are all important aspects. As a result, transformation domains, including singular value segmentation (SVD), discrete cosine transform (DCT), and discrete wave transform (DWT), are frequently employed. The spatial domain is less reliable than that of the DCT type, particularly versus processes like brightening, softening, and noise reduction filtering [15]. In addition, DWT is growing in popularity given its ability to facilitate transformation, which greatly strengthens the security of watermarked digital images. The DWT domain divides the image into several resolution levels and a starting set of processes ranging from highest to lowest resolution [16]. The measure of durability is thus increased by masking watermarks using greater intensity during digital images. Currently, SVD is broadly applied to the watermarking of digital images. SVD maintains the covered image's visualization, as well as its sturdiness against numerous forms of attack [17, 18]. As computer systems and servers continue to come closer to utilizing human-level skills, the fields of machine learning (ML) and learning techniques have also developed in recent years. Today, companies have already begun seeking opportunities to leverage their enormous datasets, such as a test platform for developing algorithms that can engage with the environment in much more practical ways and retrieve heretofore undiscovered insights. Numerous difficulties in speech signal analysis, image processing, computational linguistics, and natural language processing (NLP) can be solved with deep learning- (DL-) based neural network (NN) methods [19–22].

In addition, the convolutional neural network (CNN), a form of deep neural network, has already been utilized, largely for image recognition, fragmentation, categorization, and certain other autocorrelated data analysis [23]. Noise removal from and enhanced clarity of images are two digital image processing techniques of considerable significance that can increase image quality. Neural networks have recently been used to enhance deblurring effectiveness and accuracy by establishing mappings among clear and distorted images [24–27]. CNN can obtain successful results for image denoising, achieving promising outcomes that can be attributed to its massive modeling capability and significant breakthroughs in the training process in the network and design. CNN, using a deep structure model, improves the training phase and noise removal by increasing the capability to leverage image features. Batch normalization and the rectified linear unit (RLU) represent two learning strategies for developing and training CNN, which have made significant progress. Given that an embedded watermark is essentially a chain of noise implanted in an image, this form of noise removal could likely damage the image. Because it extracts the initial value for every pixel contained in a given image, image enhancement and noise removal present serious opportunities for attacks on digitized embedded watermark images [28–30]. The effectiveness of a fully convolutional neural network (FCNN) over watermarked images was investigated in the present study. We sought to determine whether the normalization of denoising could be utilized as a unique sort of attack through the computerized digital watermarking of images by comparing it to the SS and STDM watermarking approaches.

The digital watermarking images have various forms of attacks, including loss compression, additive noise, geometric deformation, and background subtraction attacks, which may potentially influence watermarked digital images [31, 32]. Salt-and-pepper noise and multiplicative Gaussian noise attacks are the most popular noises that threaten digital watermarking images. For a simple 8-bit grayscale image, salt-and-pepper noises modify the value of each pixel into 0 or 255 (white and white), while cumulative Gaussian noises lower the quality of an image's visual appearance. Image-filtering attacks using averaging, Wiener, median, and Gaussian filtration can effectively erase a watermark that was embedded in a digital image. The median filter is defined as a nonlinear adaptive filtering approach that maintains an image's boundaries while eliminating noise. The Wiener filter is widely used to remove blur from images. The averaging filter lowers brightness variance among pixels by substituting every pixel's value well with the weighted mean of its own neighbors and itself. The Gaussian filter is commonly adopted to blur images while reducing intensity and distortion. Geometric attacks can cause image distortions generated through processes including scaling, rotating, clipping, and translating [33, 34]. Geometric attacks are divided into two categories: local and global. Local geometric threats, namely, chopping attacks, influence parts of the image, whereas global geometric attacks, like rotational and scale attacks, disrupt every pixel in an image. To enhance the durability of different types of geometric attacks, numerous methods have been proposed.

Li et al. [35] proposed a wavelet tree quantization-based blind image using a stenographic approach to improve resistance against geometric distortions, including rotating, resizing, and cutting. Focusing mostly on SVD and the distribution of DWT, Liu et al. [36] proposed scalable multiscale full-band-based image watermarking. Cropping and rotating attacks are not a problem for this approach. Li [37] developed a computer-created hologram-based image watermarking system that is resistant to cryptographic attacks such as translating, rotating, chopping, tilting, and resizing. He et al. [38] suggested a geometrically robust image watermarking technique depending on histogram manipulation, encompassing rotating, cropping, and resizing as well as translation bouts. Regarding the mitigation of geometrical attack, Fazli and Moeini [39] have provided a durable-image watermarking system. There are a number of methods used to embed a host image, such as DWT and SVD methods, as well as DCT [40–45]. Furthermore, some authors have used discrete Fourier transform (DFT) [12–14] to embed host images, proposed DWT [46–48], and presented singular value SVD [49–51]. This technique improves the durability of resizing, translating, and rotating attacks. Two additional types of attacks—JPEG image compression and constant gain attack (CGA)—can damage a watermarked image's watermark information. A CGA attack was used to obtain factors to modify the luminance and blackness of watermarked digital images. Li et al. [52] used a perception-based model to increase the STDM watermarking system's resistance to JPEG compression. In another study presented by Lin et al. [53], the authors enhanced a type of JPEG compression that has been adopted in image watermarking systems. Recently, the CNN technique has been used to develop image priors for removing noise. For image denoising, Zhang et al. [54] developed a deep network CNN (DnCNN) framework that is able to contain convolutional kernels of the size 3∗3 for image watermark attack detection. Such a deep network is made up of various layers with distinct convolutional structures. Convolution+Relu are used in the initial layer (first layer), convolution+BatchNorm+Relu are adopted in the hidden layer, and simply the Pooling layer is used in the final layer, whereby the downsampling task is performed. The networks of 17–20 layers learned for blinded denoising with specified levels of noise using cumulative Gaussian denoising surpassed the WNNM [55] and BM3D [56] noise filtering algorithms. Using such algorithms could significantly improve the detection of watermarked image attacks. Zhang et al. [57] presented a new technology called FFDNet, which can address a broad range of excessive levels of noise. FFDNet uses a CNN model similar to that of DnCNN for quick and appropriate denoising; however, this method does not allow for the precise identification of noises. In this design, a bidirectional downsampling operator and adjustable noise-level mapping transfer the image as input into four images to be used in the CNN layers. One of biggest challenges to analyzing watermarked images is invisibility and robustness. A number of studies have sought to find a tradeoff or balance between invisibility and robustness [58], including proposing an artificial bee colony (ABC) [59–61], employing a firefly algorithm [62], and using particle swarm optimization (PSO) [63, 64]. The main contributions of the present study are as follows:

1. We have developed a hybrid model to detect various types of attacks for enhancing watermarked images
2. In the proposed system, we have used our own watermarked images to verify the ability of the proposed system
3. The proposed system was evaluated and tested with different types of evaluation metrics
4. We have applied a scaling factor to measure invisibility–robustness that is used to balance the relationship between these two characteristics, which can help end users control the watermarked images

## 2. Materials and Methods

Numerous noise sources continue to impact the visibility of digital images. White noise and additive white Gaussian noise (AWGN) represent two types of noise that can be handled by the proposed system.  Figure 1 displays the framework of the proposed system to enhance invisibility and robustness on watermarked images to detect various types of attacks.

### 2.1. Embedding Watermark Images

Figure 2 shows the steps necessary to embed a host image to create watermarked images. The procedure to embed watermark images is as follows:

1. Select the hosting watermark images
2. Apply the DWT method to the original image
3. Apply the SVD method to *LL*_*m*_ of original and watermark images
4. Use the singular value to compute with single factor *α*
5. Use the SVD to generate the watermark *LL*_*m*_

### 2.2. Discrete Wavelet Transformation (DWT) Method

DWT is a well-known statistical transformation with a wide range of application-based systems that can be implemented in engineering and science [35]. It delivers energy-efficient input image representation and also has a significant impact and durability on various image recognition attacks in watermark images [17]. DWT divides the original digital image into four spectral bands: low-high (LH), low-low, high-low (HL), and high-high (HH). After the first phase of DWT, the majority of the data details in the input images are focused within the low-low subband. The wave theory allows for even further subdivision until the width of the bands meets the watermark image specifications. In particular, when compared to other subbands, LL appears to perform better against attacks such as filtering and compressing [28, 30]. Because of this performance, the LL subband can be an attractive option for powerful watermarking [37].

### 2.3. Singular Value Decomposition (SVD) Method

In this method, singular values are differentiated throughout the structure of the symmetric matrix when SVD disintegrates the homogeneous matrix, thus generating three specific matrices [46]. Underneath the matrix decomposition, the three deconstructed matrices include the left single matrix *U*, single matrix *S*, and right single matrix *V*. Assuming *Y* represents a symmetric matrix, the SVD is calculated in the following equation:

(1) $$\begin{array}{c} USV^{T}=\text{SVD}\left(Y\right), \end{array}$$

where *VV*^*T*^ = *I*_*n*_ and *UU*^*T*^ = *I*_*n*_. The column elements of *U* are represented by the orthonormal eigenvectors of *YY*^*T*^. These orthonormal eigenvectors are also denoted by columns *V* in the *Y*^*T*^*Y* matrix, and *S* is indicated as a diagonal matrix, which encompasses the square roots of the eigenvalues determined from *U* or *Vi*n the descendant direction. If *r*(*r* ≤ *n*) refers to the standing of matrix *Y*, then the factors of the diagonal matrix *S* can be represented as a relative association in equation (2), and matrix *Y* is expressed in equation (3):

(2) $$\begin{array}{c} \sigma_{1}\geq \sigma_{2}\geq \cdots \geq \sigma_{r}\geq \sigma_{r+1}=\sigma_{r+2}=\cdots =\sigma_{n}=0, \end{array}$$

(3) $$\begin{array}{c} Y=\overset{r}{\underset{i=1}{\sum }}\sigma_{i}\mu_{i}v_{i}, \end{array}$$

where *v*_*i*_, *μ*_*i*_, and *i*_*th*_ represent the eigenvector of *V* and *U* and *σ*_*i*_ indicates the *i*_*th*_ singular value. Throughout this work, the singular value of the watermark is integrated through the host image by such an appropriate magnification factor, and the singular value of the watermark is incorporated further into the host image by using sufficient scaling factor. The invisibility and resilience of the watermarking process are two important aspects of this process. Because the scaling factor remains insufficient, the accurate effectiveness of the suggested method must be optimized. As a result, an optimized algorithm is needed to achieve the maximum relationship between invisibility and resilience of a watermark image.

### 2.4. Feature Extraction of Watermark Images

Feature extraction is crucial for identifying significant features in the watermark image. The image mage *I* and the output of the image are referred to as the watermarking image *m*^∗^. Procedure steps to extract the features from inputted watermark images are presented in Figure 3. The procedure steps of the proposed system to extract significant features are as follows:

1. Setup image *I*
2. Use DWT to decompose image into four levels: *LL*_*m*_, *HH*_*m*_, *LH*_*m*_, and *HL*_*m*_
3. Apply SVD to *HH*_*m*_

(4) $$\begin{array}{c} HU^{*}\;HSb_{m}^{*}HV_{m}^{*}=\text{SVD}\left(HH_{m}\right), \end{array}$$

(5) $$\begin{array}{c} \;S_{m}^{*}=\frac{HSb_{m}^{*}-HS_{m}^{*}}{\alpha }. \end{array}$$

*S*_*m*_^∗^ is used to extract the singular value; we have used the inverse SVD method to reconstruct the watermarking image *M*^∗^.

### 2.5. Measurement Performance

Three evaluation metrics, namely, peak signal-to-noise ratio (PSNR) and structural similarity index measure (SSIM), were employed to determine invisibility. To evaluate robustness, the normalization correlation (NC) was applied:

(6) $$\begin{array}{c} \text{PSNR}\left(C,C^{*}\right)=101g\frac{C_{\max}^{2}}{\text{MSE}}, \end{array}$$

(7) $$\begin{array}{c} \text{MSE}=\frac{1}{M^{2}}\overset{M}{\underset{i=1}{\sum }}\;\overset{M}{\underset{j=1}{\sum }}{\left(C_{i}j-C_{i}^{*},j\right)}^{2}, \end{array}$$

(8) $$\begin{array}{c} \text{SSIM}\left(C,C^{*}\right)=\frac{\mu c\mu c^{*}+d_{1}}{\mu^{2}c+\mu^{2}c+d_{1}}.\frac{\sigma cc^{*}+d_{2}}{\sigma^{2}c+\sigma^{2}c*+d_{2}}, \end{array}$$

(9) $$\begin{array}{c} NC=\frac{\sum_{I=1}^{N}\sum_{J=1}^{N}W_{i,j}w_{i,j}^{*}}{\sqrt{\sum_{i=1}^{N}\sum_{j=1}^{N}w_{i,j}^{2}}\;\sqrt{\sum_{i=1}^{N}\sum_{j=1}^{N}w_{i,j}^{2}}\;}, \end{array}$$

wherein *C* is the host image, MSE is the mean square error, *M* is the output watermark, *C*_*i*_ is the host image, *C*_*j*_ is the watermark image, *μc* is the average values of the host image, and *σ*^2^ is the variance.

## 3. Experimental Results

In this section, the results of the watermark algorithm are presented, and the invisibility and robustness of watermark images are analyzed using the DWT and SVD algorithms. The results of the proposed system were used to determine the scaling factor of watermarks of different sizes by employing PSNR, SSIM, and NC.

### 3.1. Environment of the Proposed System

Table 1 shows the proposed system requirements in terms of hardware and software.

### 3.2. Dataset

In this experiment, two images were used, one of a lion and one of a cameraman, to test the proposed system, and the grayscales of the images were 512 × 512 and 256 × 256, respectively.  Figure 4 shows the two images used to examine the proposed system.

The performance of the proposed system was evaluated by various attacks, such as filter, cropping, rescaling, histogram equalization, sharpening, noise, compression, motion blur, and rotation attacks. The table summarizes the various attacks.

### 3.3. Results

#### 3.3.1. Scaling Factor of Watermarks

The scaling factor is calculated by using multiple sizes to require being taken back to OEF. In the proposed system, the host image lion (512 × 512) and the watermark cameraman image (256 × 256) are applied to determine optimal scaling by observing the relationship between the scaling factor and significant parameter values, controlling the invisibility and robustness of watermarked images for identifying various types of attacks. The scaling factors of various parameters for detecting attacks are presented by using the NC metric (Figure 5). The scaling factors of attack values [0.02-0.2] are noted, whereas the *y*-axis NC (*W*, *W*∗) presents watermark images and *x*-axis scaling factors *α*.

Figure 6 shows the scaling factors of the various attacks using the PSNR metric. The *y*-axis represents the values of PSNR, and it was observed that the values of motion blur and average filter were very low. The *x*-axis shows the scaling factors of all attacks.

The scaling factors of the SSIM metrics are presented in Figure 7. Regarding the scaling factor values of all attacks (*y-*axis) ranging between 0 and 0.9, it was observed that the Gaussian noise resulted in less scaling compared to various types of attacks.

#### 3.3.2. Results and Discussion

We examined the target watermark images to identify various attack types, including Gaussian low-pass filter, median, Gaussian noise, salt-and-pepper noise, speckle noise compression, sharpening, histogram equalization, average filter, and motion blur attacks, as well as no attack. The evaluation metrics were applied to measure the parameter values, such as SSIM and PSNR used to analyze the watermarked images after the injection of attacks; moreover, NC was employed to test the robustness between the hosting image and watermark image after being subjected to various attacks.

Table 2 shows the results of the proposed system by employing the NC metric to determine the level of robustness of the parameter values of the attacked watermark images. The proposed system achieved good robustness for enhancing the quality of embedded images: no attacks (98.74%), salt-and-pepper noise (98.24%), and speckle noise (98.31%), whereas NC decreased values with motion blur (70.77%). Overall, the system was shown to improve watermarked images in terms of filtering all types of attacks.  Figure 8 displays the results of the DWT-SVD algorithm to extract significant values from watermarked images after applying attacks. It was observed that the values of NC were superior for most attacks.

Table 3 shows the results of the proposed system in terms of the relationship between the level of invisibility of the embedded image and determining the likelihood of watermark attacks. The proposed system achieved optimal quality of grayscale watermarked image attack on no attack (PSNR = 52.70, SSIM = 99.99%). The system achieved lower quality invisibility in terms of watermarked image histogram equalization (PSNR = 14.04) and Gaussian noise (SSIM = 70.53%).  Figure 9 shows the invisibility performance of extracting attacks from watermarked images using PSNR and SSIM metrics. It was noted that watermarked images have good invisibility.

When invisibility is found, robustness must be analyzed and evaluated; therefore, it is crucial to confirm the robustness of embedded images to identify various types of attacks and thus enhance the watermarked images in response. The proposed system was used to measure the invisibility and robustness for obtaining good results in managing all types of watermarked attacks.

#### 3.3.3. Comparison Results

All parameters were evaluated to examine the attacks static, and we applied the proposed system dynamic to test the efficiency and effectiveness of the proposed system.  Figure 10 shows the testing phase of the proposed system to check the level of robustness in the quality of the watermarked images. We selected parameters with different sizes of images to examine our proposed system. Furthermore, when the proposed system of DWT-SVD was compared to other systems, it was observed that the results from the proposed system achieved high accuracy in detecting various watermarked attacks. In the present research, various attacks were imposed on the host image to obtain optimal performance.

The research article (Makram et al., 2021) applied a deep learning model to measure the level of robustness of watermarked images after applying attacks, with the authors using six attacks, namely, salt-and-pepper, Gaussian filtering, median filtering, average filtering, and FCNNDA. However, in the proposed research, 11 attacks were considered to enhance the watered images. We compared the results of the proposed system to the existing system in the case of some attacks. The comparison results of Makram et al. (2021) against the proposed research are presented in Table 4. It was observed that the results of the proposed system were superior.

Table 5 shows results of the proposed system against the existing system; in (Arora et al., 2018), the researchers have used the DWT method. The existing system used histogram equalization, salt-and-pepper noise, sharpening, and Gaussian noise attacks to examine their system. It is observed that the proposed system has achieved better than their DWT method.

Furthermore, the results of our proposed system was compared with SVD, which is the existing mode of Joseph et al. (2013); four attacks, namely, histogram equalization, salt-and-pepper noise, sharpening, and Gaussian noise attacks, are presented in Table 6. It is noted that the proposed system is superior.

## 4. Conclusion

At present, information can be duplicated easily due to the interactive nature of the digital communication of multimedia data. In this paper, we developed a digital watermark method using DWT-SVD that analyzes various types of watermark attacks. This approach was designed to determine the relationship between invisibility and robustness using scaling factors. The focus of this research was the ability to embed and extract various attacks on watermarked images without restrictions on the host or the watermarked images and, furthermore, to enhance this ability by sufficiently monitoring the invisibility and robustness. Some important aspects of the present study are as follows:

- DWT was used to embed the host image into watermarked images to test the proposed system
- DWT-SVD was applied to extract various types of significant features to identify all watermark attacks
- We used three evaluation metrics, namely, SSIM, PSNR, and NC, to examine the obtained results from the proposed system. The SSIM and PSNR metrics were applied to evaluate the invisibility of the watermarked images, and NC was used to measure the robustness of watermarked images in terms of analyzing the attacks
- The empirical results showed the excellent performance of the proposed system in measuring all types of attacks employed in the study
- The results of the proposed system were compared with state-of-the art works, and it was observed that the proposed system showed better performance

Consequently, we believe the proposed system would be helpful to the field of watermarking for managing digital images, as it permits the embedding and extraction of watermarked images without limitations on the host image and WM information. The proposed system can help to enhance and control invisibility and robustness to achieve optimal performance in response to a variety of attacks.

## Figures and Tables

**Figure 1:** Proposed system.

**Figure 2:** The watermark embedding procedure.

**Figure 3:** Feature extracting procedure.

**Figure 4:** Emended watermark images: (a) own image and (b) standard image.

**Figure 5:** Scaling factors of various parameters by using NC: (a) lion image and (b) Elaine image.

**Figure 6:** PSNR scaling factors: (a) lion image and (b) Elaine image.

**Figure 7:** SSIM scaling factors: (a) lion image and b) Elaine image.

**Figure 8:** Watermarked images after applying different attack types: (a) lion image and b) Elaine image.

**Figure 9:** Performance of proposed system to extract attacks from watermarked images with respect to invisibility: (a) lion image and (b) Elaine image.

**Figure 10:** Parameters with different types of attacks with respect to NC values: (a) lion image and (b) Elaine image.

**Table 1:** System requirements.

Hardware	Software
RAM 8 GB	MATLAB R2020a
CPU I7	Windows 10

**Table 2:** Performance of the DWT-SVD method to identify robustness and quality of watermarked images.

	Lion image	Lena image
Attacks	NC	0.9975
No attack	0.9874	0.8243
Gaussian low-pass filter	0.9028	0.9246
Median	0.958	0.9755
Gaussian noise	0.9599	0.9937
Salt-and-pepper noise	0.9824	0.9919
Speckle noise	0.9831	0.9942
Compression	0.96255	99.664
Sharpening	0.9334	0.9024
Histogram equalization	93.14	0.9341
Average filter	0.90063	0.822
Motion blur	0.70774	0.6648

**Table 3:** Performance of the DWT-SVD method to find invisibility and quality of watermarked images.

Attacks	Lion image		Lena image	
	PSNR	SSIM	PSNR	SSIM
No attack	52.70	0.99989	47.93	0.9998
Gaussian low-pass filter	38.25	096.774	33.74	0.9148
Median	38.8989	0.9719	35.23	0.9227
Gaussian noise	29.956	0.7053	29.92	0.694
Salt-and-pepper noise	35.4581	0.9739	35.317	0.9736
Speckle noise	37.85	0.9450	35.336	0.8756
Compression	38.85	0.9645	35.52	0.9184
Sharpening	38.88	0.9813	37.86	0.9359
Histogram equalization	14.04	0.7492	34.966	0.96405
Average filter	38.12	96.68	19.117	0.8528
Motion blur	31.75	0.85.622	33.62	0.8528

**Table 4:** Comparison results of the proposed system against an existing study [50].

Proposed system			Existing system	
Attacks	NC	SSIM	NC	SIMM
Median	0.958	0.9719	0.966	0.878
Salt-and-pepper noise	0.9824	0.9739	0.890	0.612
Average filter	0.90063	96.68	0.820	0.418

**Table 5:** Comparison results of the proposed system against an existing study [65].

	Proposed system	Existing system
Attacks	NC	NC
Histogram equalization	0.958	0.5765
Salt-and-pepper noise	0.9824	0.5775
Sharpening	0.90063	0.52
Gaussian noise	0.9028	0.5512

**Table 6:** Comparison results of the proposed system against an existing study [66].

	Proposed system	Existing system
Attacks	NC	NC
Histogram equalization	0.958	0.820
Salt-and-pepper noise	0.9824	0.82
Sharpening	0.90063	0.791
Gaussian noise	0.9028	0.831

## Data Availability

The standard images are from MATLAB https://www.mathworks.com/matlabcentral/answers/263183-where-to-download-the-example-image.
